# Memristive GAN in Analog

**DOI:** 10.1038/s41598-020-62676-7

**Published:** 2020-04-03

**Authors:** O. Krestinskaya, B. Choubey, A. P. James

**Affiliations:** 1 Unaffiliated, Nur-Sultan, Kazakhstan; 2 Analogue Circuits and Image Sensors, Siegen University, Siegen, 57080 Germany; 3 Artificial General Intelligence and Neuromorphic Systems (NeuroAGI), Indian Institute of Information Technology and Management - Kerala, Trivandrum, Kerala 695584 India

**Keywords:** Electrical and electronic engineering, Electronic and spintronic devices

## Abstract

Generative Adversarial Network (GAN) requires extensive computing resources making its implementation in edge devices with conventional microprocessor hardware a slow and difficult, if not impossible task. In this paper, we propose to accelerate these intensive neural computations using memristive neural networks in analog domain. The implementation of Analog Memristive Deep Convolutional GAN (AM-DCGAN) using Generator as deconvolutional and Discriminator as convolutional memristive neural network is presented. The system is simulated at circuit level with 1.7 million memristor devices taking into account memristor non-idealities, device and circuit parameters. The design is modular with crossbar arrays having a minimum average power consumption per neural computation of 47nW. The design exclusively uses the principles of neural network dropouts resulting in regularization and lowering the power consumption. The SPICE level simulation of GAN is performed with 0.18 *μ*m CMOS technology and WO_*x*_ memristive devices with *R*_*ON*_ = 40 kΩ and *R*_*OFF*_ = 250 kΩ, threshold voltage 0.8 V and write voltage at 1.0 V.

## Introduction

Intelligent near-sensor analog computing requires integration of neural co-processor unit next to the sensing unit. The analog memristive neuromorphic circuits^1^ can integrate complex neural networks and learning systems to edge devices and sensors due to the advantages offered by memristors in area efficiency, non-volatility, programmability, high switching speeds, and low power requirements. Generative Adversarial Network (GAN) is a well known computationally complex neural network architecture for generating new patterns that requires significant computational resources in software implementations as well as large amount of data for training^2^. This makes its implementation in edge devices with conventional microprocessor hardware a slow and difficult task. Recently, there have been several works proposing to accelerate GAN and implement the generative networks on FPGA^3,4^ and digital CMOS circuits^5^. These solutions have high power consumption and on-chip area for implementing within a edge device. The implementation of GAN on edge devices will eliminate the requirement of sending large amount of data collected by a sensor (e.g. in a camera) to a server for processing, which can speed up the GAN training on low power devices, where on-chip area, memory and power consumption is limited.

The application of memristive devices for GAN can be a promising solution for near-sensor edge computing due to small on-chip area and low power consumption. Previously, memristive devices have been used for accelerating the vector-matrix multiplication operations in the neural networks and learning systems on hardware^6^. Recently, a 128 × 64 reconfigurable hafnium oxide memristive crossbar has been tested for analogue vector-matrix multiplication with high device yield and high state retention for image processing applications^7^. An integrated 128 × 64 1T1R crossbar array has been used in a Long-Short Term Memory (LSTM) network with software-based implementation of the activation functions for regression and classification tasks^8^. Reinforcement learning has also been tested on analogue memristor arrays in 3-layer network using hybrid mixed-signal system^9^. The in-situ training of convolutional neural network (CNN) using tantalum oxide memristive crossbars and digital and software-based activations and processing circuits has been shown recently^10^. Finally, the fully integrated reconfigurable memristor chip with a 54 × 108 WO_*x*_ memristor array, digital processing circuits and OpenRISC has been reported^11^.

The application of memristive crossbars to accelerate software-based GANs has also been explored^12,13^, and the intrinsic random noises of ReRAM devices have been used as a random input to GAN to improve the diversity of the generated numbers^14^. In addition, several digital implementations of GAN accelerators with conventional digital architectures and ReRAM crossbars have been demonstrated recently^15–17^. However, the circuit level implementation of analog GAN architecture for near-sensor on-edge processing has not been proposed yet. In this work, we present a Deep Convolutional Generative Adversarial Network (GAN) that can be integrated as a near-sensor intelligent computing solution.

We present a fully analog hardware design of Deep Convolutional GAN (DCGAN)^18^ based on CMOS-memristive convolutional and deconvolutional networks simulated using 180 nm CMOS technology and WO_x_ memristive devices^19^, and propose to accelerate the computationally intensive GAN using memristive neural networks in analog domain to be applicable to implement on edge devices. The main contributions of the paper are the following: (1) the design and circuit level implementation of a Deep Convolutional Generative Adversarial Network with memristive crossbar arrays having 1.7 million memristor devices, (2) a scalable design that provides high robustness to conductance variability, circuit parasitics and device non-idealities, which is verified in the paper, and (3) as the presented architecture is analog, it can be integrated into the chip for near-sensor processing without the analog to digital conversion for both training and image generation. This can increase the processing and training speed and reduce the power consumption, comparing to traditional CPU- and GPU-based GAN processing^20^, making the architecture applicable for edge processing.

## The proposed GAN architecture

### Overall architecture

GAN utilizes two neural networks with competitive learning approach: (1) a Generator to produce a new data from the input noise and (2) a Discriminator to discriminate this new data from the training data^2,18^. Figure 1(a) illustrates a hardware implementation of the proposed Analog Memristive Deep Convolutional Generative Adversarial Network (AM-DCGAN). The proposed implementation is inspired by DCGAN algorithm^18^. While the original GAN algorithm is complex and may require batch normalization between layers and max-pooing operation to introduce non-linearity to the system, in the proposed hardware implementation the normalization is not considered and mean-pooling (average-pooling) is used to ensure the simplified implementation in analog domain. For the simple applications like MNIST, the pooling layer is not necessary and the architecture can perform well without it; however, for more complex problems and RGB images, the pooling layer is required. The architecture is applicable for small-scale problems, like handwritten digits generation illustrated in the results section, and shows the proof of concept that GAN can be implemented using analog CMOS-memristive circuits.

**Figure 1:** (**a**) Total Analog Memristive Deep Convolutional Generative Adversarial Network (AM-DCGAN) architecture. (**b**) Example of generated images after MNIST training. (**c**) Generator architecture consisting of Deconvolutional Neural Network (DCNN). (**d**) Discriminator architecture consisting of Convolutional Neural Network (CNN).

In the AM-DCGAN architecture shown in Fig. 1, the Generator Network has been implemented as a Memristive Deconvolutional Neural Network (DCNN). The Discriminator Network, on the other hand, is a Memristive Convolutional Neural Network (CNN). During training of these neural networks, the Generator produces the fake images from input noise, while the Discriminator is trained to identify whether the produced image is fake or real using supervised training method. The Discriminator acts as a binary classifier producing a single output. An example of generated images after training this network on MNIST handwritten digit database^21^ is illustrated in Fig. 1(b). The AM-DCGAN architecture can be integrated to the image sensor to read the real images directly from the sensor without the application of analog-to-digital converter (ADC). To remove thermal noise and fixed pattern noise in the analog domain in such system, subtracting and memory circuits can be utilized^22^. In this work, training with Adam optimizer^23^ and binary cross-entropy loss function is used for error calculation and update of memristive devices. The training unit performing error propagation and weight updated can also be implemented on-chip. However, such chip would need to be implemented in digital as the endurance of memristors are limited, with repeated writes causing faster aging, and would end up reducing the reliability of inference operation.

Deconvolution and Convolution operations in these circuits are performed using memristive crossbar based dot product multiplication. In the Generator block containing *k* layers, as shown in Fig. 1(c), the input noise is provided to the first deconvolutional layer. This and subsequent layers consist of a number of deconvolution filters, F. The filter outputs are fed to a normalization layer with rectifier linear unit (ReLU) circuits, which outputs only positive inputs. To enhance the training of GAN, especially for complex datasets, the leaky ReLU (LeakyReLU) activation function should be used (circuit level implementation of both is shown in Methods section). This deconvolution process is performed several times to achieve the desired size of the image. In the last layer of the Generator, a hyperbolic tangent (tanh) activation function is used instead of ReLU. The input to this last layer can be either positive or negative. Therefore, the memristive filter with both positive and negative weight (represented by 2 memristors) are used; while for all the previous layers the filters with only positive weights (containing 1 memristor) is enough for simple applications to reduce the complexity of the architecture. However, the performance of the system with both positive and negative weights in both convolutional and deconvolutional filters is still better.

Figure 1(d) shows a CNN based Discriminator. It consists of several memristive convolutional layers with convolutional filters (F), mean pooling layers with memristive mean filter (M) and a memristive dense network. The convolutional layer output is fed to the ReLU activation function followed by the mean pooling operation. While for MNIST application shown in this work, the pooling operation is not required and can be removed without compromising on the performance of the system, pooling is necessary for more complex applications. Therefore, in this system we show the memristive mean-pooling filters that can reduce the complexity of analog CNN, comparing to the implementation of having a max-pooling operation. The mean output is then fed to the next convolution layer. After the last convolutional layer, the output image is processed by the dense network, which is another memristive neural network; however with only one output depicting if the image is “fake” or “real”. The circuit level implementation of the components of the architecture is illustrate in the Methods section.

### Circuit components

Individual elements of two networks are designed using a typical 180nm CMOS process. The circuits are shown in Fig. 2, with the design parameters presented in Fig. 2(l). Other system components, including the activation functions, are designed using analog CMOS circuits as shown in Fig. 2.

**Figure 2:** Circuit components used in AM-DCGAN: (**a**) Deconvolution/convolution filter (F), (**b**) Rectifier linear unit (ReLu) and LeakyReLU circuits, (**c**) Deconvolution/convolution filter with sign control mechanism (Fs), (**d**) Hyperbolic tangent (tanh), (**e**) Mean pooling Filter (M) from CNN, (**f**) Operational Amplifier (OpAmp), (**g**) Weight Sign Switch (WSS) circuit, (**h**) current to voltage converter (IVC), (**i**) Control Switch (CS), (**k**) Analog Sample and Hold circuit, and (**l**) circuit parameters.

#### Convolution, deconvolution and mean filters

Convolution and deconvolution filters are realized as a single column of small memristive crossbars, as shown in shown in Fig. 2(a). The weights represented by the conductance of memristive devices in these filters are trained during the training stage. In the deconvolution operation, the crossbars can be of different sizes depending on the input image and required upsampling operation.

The filter of Fig. 2(a) is used only for positive synapses as is required in majority of the layers of CNN and DCNN for simple applications (like MNIST). This reduces the complexity of the circuits by removing the requirement of placing an OpAmp based current to voltage converter after each convolutional filter. However, for more complex databases, both positive and negative synapses are required, otherwise, the performance will be deteriorated. The input to the filter *V*_*in*_ is normalized to the range [−*V*_*th*_, *V*_*th*_], where *V*_*th*_ is a threshold voltage of the memristor. The output of each crossbar *V*_*outF*_ is read across the load memristor or a set of parallel load memristors, when the minimum resistance of the memristor is higher than the required load, as illustrated in Fig. 2(a). The output voltage *V*_*outF*_ is shown in Eq. (1), where *R*_*L*_ is a total load resistance. When *R*_*L*_ = *R*_*L*1_ = *R*_*L*2_ = . . . = *R*_*Lk*_, *R*_*L*_ = *R*_*Lk*_/*k*, where *k* is a number of memristors in parallel.

1 $${V}_{outF}=\frac{{\sum }_{x=1}^{N}\frac{{V}_{inx}}{{R}_{x}}}{\frac{1}{{R}_{L}}+{\sum }_{x=1}^{N}\frac{1}{{R}_{x}}}\,{\rm{,\; where}}\,{R}_{L}=\frac{1}{{R}_{L1}}+\frac{1}{{R}_{L2}}+\ldots +\frac{1}{{R}_{Lk}}$$

As this method utilises the voltage divider principle, the normalization of voltages between *V*_*outF*−*H*_ and *V*_*outF*−*L*_ (which are the highest and lowest outputs of *V*_*outF*_) is performed automatically. This also prevents the output voltage from exceeding the maximum filter input *V*_*in*_ (or *V*_*th*_). Our design contains four *R*_*L*_*k* memristors in parallel. This memristors replace the necessity to put load resistor to read the voltage across it and reduce on-chip area. In the proposed design, the total load resistance should be equal to 1 *k*Ω. As for WO_*x*_ memristors, *R*_*ON*_ = 40 *k*Ω, to create the total load of 10 *k*Ω, four devices in parallel are required. Depending on the memristor material, the number of these devices may vary. In addition, of the on-chip area of the architecture is not a critical aspect, load resistors can be used instead of memrsitors to reduce the fabrication complexity.

The last block of the Generator circuit, however, is a hyperbolic tangent activation function requiring both positive and negative inputs. Hence, the last deconvolutional layer utilises a different filter with positive and negative weights in memristive structures. Such filters can be used in all the convolutional and deconvolutional layers of the architecture, when it is necessary to enhance the performance of the system for more complex applications. In this filter (Fs), shown in Fig. 2(c), negative synapses are created using two memristors and an OpAmp-based subtractor^1^. However, rather than using conventional method with a current-to-voltage converter, we read voltages across the load memristors. To implement positive synapses, *G*^−^ is set to *R*_*OFF*_, while *G*^+^ varies according to the required weight value. To create negative synapses, *G*^−^ vary and *G*^+^ is set to *R*_*OFF*_. This method, while being a very efficient circuit, also allows us to obtain weight *w* = 0. The tangent circuit (tanh, shown in Fig. 2(d)) provides a “hard” tangent function. Hence, the low output voltage of the filter ensures the limits of the the input to the tanh circuit. The OpAmp used has two differential and one common gain stages with indirect compensation technique, is shown in Fig. 2(f)^24^. Depending on the *R*_*ON*_/*R*_*OFF*_ ratio of the devices and mapping method, an additional amplification may be required for *V*_*outF*_ and ${V}_{out{F}^{{\prime} }}$.

The memristive mean-pooling filters used in the Discriminator are shown in Fig. 2(e). They consist of *M* memristors set to maximum resistance *R*_*OFF*_ to limit the current flowing through the memristor and in turn overall power consumption. The mean filters are illustrated separately rather than is a strided convolution operation with convolution filters to emphasize that these filters are not trainable and always set to *R*_*OFF*_. The memristive mean-pooling filters are used to reduce the on-chip area of the architecture, comparing to max-pooling operation. These filters are optional for the MNIST application, as the problem is simple and pooling can be avoided. However, such filters will be useful when training the architecture to generate more complex RGB images.

#### Activation functions

The activation functions used in AM-DCGAN are either ReLU/LeakyReLU, as shown in Fig. 2(b) or hyperbolic tangent (tanh), as shown in Fig. 2(d). The ReLU circuit is based on a transmission gate. The input voltage is applied to the inverter *M*_1_/*M*_2_ and transmission gate *M*_7_/*M*_8_. The inverters are designed with a threshold *V*_*thReLU*_ = 0*V*. Depending on the sign of the input, if the transmission gate is on, the voltage *V*_*inR*_ is passed to the output *V*_*outR*_ = *V*_*inR*_. If the transmission gate is off, *V*_*outR*_ = 0, due to action of the second transmission gate *M*_9_/*M*_10_. The way to change the ReLU to LeakyReLU is proposed in Fig. 2(b). Instead of connecting the transmission gate *M*_9_/*M*_10_ to the ground for the case of negative input, it is connected to voltage divider *R*_*LR*1_-*R*_*LR*2_ which reduces the input voltage fro negative case by the ratio *R*_*LR*2_/*R*_*LR*1_. In this work, this ratio is set up to 100/400 to satisfy LeakyReLU equation *y* = *max*(0.2*x*, *x*). The “hard” hyperbolic tangent (tanh) (Fig. 2(d)) is also implemented with two adjusted inverters with parameters shown in Fig. 2(l). The “hard” tanh function is selected due to small on-chip area and power consumption comparing to traditional tanh implementation^25^.

#### Dense network

The dense network in the discriminator is a conventional memristive neural network with ReLU activation function in the hidden layers and linear activation function in the output layer. The sign of memristive weights in the dense layer is controlled by the sign crossbar, which stores in the sign of each memristor. The output from the main crossbar is read sequentially one column at a time. At the same time, a row of the sign crossbar corresponding to the particular column of the main crossbar is activated. The output of the sign crossbar is controlled by the weight sign switch (WSS), which inverts the input voltage applied to the main crossbar, instead of introducing the negative weights to memristors. The sequential processing in the dense layer crossbar is controlled by the control switches (CS) using two transistors. The output current from the column is converted to voltage by an OpAmp based current to voltage converter (IVC) and processed with ReLU function. As the crossbar columns in the dense layer are processed sequentially, the voltage signal is retained using conventional Analog Sample and Hold (SH) circuit shown in Fig. 2(k). The SH circuit contains sample and hold part and two voltage buffers to reduce the effect of the other system components on the sampled signal. The parameters of SH circuit are adjusted for *ns* operation and small capacitor value (0.05*pF*) is selected. When *V*_*clk*_ is high, the input signal is sampled. The clock signal *V*_*clk*_ of SH circuit in each column is programmed to read the ReLU output at a particular time step and retain all the outputs (*V*_*clk*_ is kept high) till the “read” of the last column is finished to supply them to the second layer in parallel. In the second dense layer, the processing is performed similarly; however, the crossbar has only one output corresponding to the particular class (“fake” or “real”).

#### Weight sign switch circuit

Weight sign switch (WSS) circuit shown in Fig. 2(g) is used to control the sign of the weights by inverting input voltages applied to the crossbar. Each weight of the network is represented by two memristors: (1) from the main crossbar and (2) from the sign crossbar. The main crossbar stores only the absolute value of the weight, while the sign crossbar stores the sign of the weight in a form of *R*_*ON*_ or *R*_*OFF*_ state of the memristors. As the columns of the main crossbar in the dense network are processed sequentially, only one column is activated in the main crossbar at a time. While in the sign crossbar all the columns are activated with a single active 1T1R cell at a time, so the signs of all the weights *V*_*outS*_ are supplied to WSS in parallel, and the outputs of all WSS circuits *V*_*outWSS*_ are fed to the main crossbar. WSS acts as a comparator and either keeps the sign of the input voltage *V*_*inWSS*_ (the output of the convolution filter) or changes it. If the voltage from the sign crossbar *V*_*outS*_ exceeds the threshold of the inverter *M*_35_ − *M*_36_ in WSS, the thresholding circuit activates the sign switch *M*_41_ − *M*_44_ controlling the difference amplifier. If the sign switch is on, the difference amplifier subtracts 2*V*_*inWSS*_ from *V*_*inWSS*_. Otherwise, *V*_*outWSS*_ = −*V*_*inWSS*_, when the output of the sign switch is set to 0 *V*. Therefore, instead of introducing negative memristive weight, we change the sign of the input, if the weight is supposed to be negative.

#### Crossbar switch and current to voltage converter

The sequential processing of the crossbar columns in the dense layers is controlled by the control switches (CS) based on two transistors shown in Fig. 2(i). The bulk of the transistors in a crossbar switch is connected to the control voltages *V*_*DD*_ (for PMOS) and −*V*_*DD*_ (for NMOS), rather than to their sources. This improves the linearity of the switch and avoids the leakage current when switch is set to “off”. Nevertheless, with the increase of the number of crossbar rows connected to the transistor, the linearity of the switch decreases. In this work, the switch and following current to voltage converter (IVC) was adjusted for 784 input rows (considering the input of 28 × 28). As the switch is nonlinear, the current does not go beyond 10 mA. In an ideal case without this switch for largest possible weights and inputs, it should be about 160 mA. This hence, normalizes the current without any additional normalization circuit. For smaller number of rows, the ideal current of 25 mA is normalized to 8 mA. Nevertheless, the effect of this normalisation on the overall performance still should be investigated further. The current to voltage converter (IVC, shown in Fig. 2(h)) after the switch is adjusted to convert the current from the switch to voltage. The maximum current is converted to the threshold voltage of the memristor for further processing. This converter provides an inverted output *V*_*inv*_ as well as a non-inverted output *V*_*outIVC*_ = −*V*_*inv*_.

### Memristor non-idealities

This work focuses on the investigation of the effect of various memristor non-idealities^26–28^, such as limited number of stable resistive states, resistance variations, device failures and the device aging, on the implementation of the proposed AM-DCGAN. When limited number of stable resistive states is added, the weights are restricted between *R*_*ON*_ and *R*_*OFF*_ resistances. The intermediate states are distributed uniformly between *R*_*ON*_ and *R*_*OFF*_ to show the impact of the limited number of states.

The variation of the resistive states of the memristor are represented as Gaussian distribution *w* = *w* + *G*_*d*_(*μ* = 0, *std* = *σ*), where *w* is a normalized weight, *G*_*d*_ is a Gaussian distribution with *μ* = 0 mean and standard deviation *std* = *σ*. Figure 3(a) shows the distribution of normalized highest and lowest memristive weights for difference standard deviation (std) of Gaussian distribution, based on the variation of *R*_*ON*_ and *R*_*OFF*_ states, and corresponding difference between neighboring states for the devices with 128 stable resistive states. Based on Fig. 4(b), the architecture based on memristive devices with weight distribution with *std* = 0.04 can still produce good quality images, while Fig. 3(a) shows that the neighboring states are still close to each other. For *std* = 0.1 and *std* = 0.2, the neighboring states (0 and 1/128 in Fig. 3(a)) completely overlap, which leads to the bad quality of the generated images (Fig. 4(b)).

**Figure 3:** Memristor non-idealities: (**a**) variation of high and low resistive states with difference standard deviation (std), and (**b**) effect of device aging on high and low states.

**Figure 4:** (**a**) Effect of the number of memristive levels (stable resistive states) on the quality of the generated images. (**b**) Effect of the variability in memristive devices on the generated images. (**c**) Effect of random device failures on the generated images. (**d**) Effect of percentage of the device aging on the performance of the architecture. (**e**) Effect of hardware variation without and with cell-to-cell memristor variation on the performance of the architecture. (**f**) Effect of noise in the input images on the performance of the architecture. (**g**) Effect of the number of training iterations on the generated images.

The failure of the devices in the architecture is introduced by setting the devices to *R*_*ON*_ (when the memristor is stack in *R*_*ON*_ state), *R*_*OFF*_ (when the device is stack in *R*_*OFF*_ state) or *R* = 0 (when the connection is failed completely and the device is not conducting the current). The percentage failure in Fig. 4(c) combines all these case. For example, 1% failure of the device means that 0.25% of random memristive weights are set to *R*_*ON*_, 0.25% of random memristive weights are set to *R*_*OFF*_, and 0.5% of the devices are completely disconnected and set to 0. This method allows to illustrate a generalized scenario of memristor failures and their effect on the performance of the architecture.

Figure 3(b) shows effect of the memristor aging of the normalized *R*_*ON*_ and *R*_*OFF*_ states (highest and lowest memristive weights in the architecture). In general, memristor aging assumes the change in the resistive levels, when high resistance level *R*_*OFF*_ decreases and low resistance level *R*_*ON*_ increases, and several highest and lowest resistive states can not be reached anymore^29,30^. In the evaluation of the proposed architecture, the general case was considered, where the decrease in *R*_*OFF*_ and increase of *R*_*ON*_ are assumed to be the same. Figure 3(b) shows how the percentage of aging used in the simulation effects the highest and lowest memristive weights in the architecture. For example, in the architecture with 128 levels, the aging of 4% the aging removes 6 highest and 6 lower resistive states; while the aging of 10% cuts 13 highest and 13 lowest states.

## Results

### System level simulations

The system has been tested on handwritten digits MNIST handwritten digits database. The Generator with 3 deconvolutional layers and 128 and 64 filter of the size of 5 × 5 (25 memrsitors), and the Discriminator with 2 convolutional layer and 64 and 128 filters of the size of 5 × 5 and single dense layer are implemented. To understand the effect of variability and limited number of stable resistive states of memristive devices, further simulations were carried out with the same database. Figure 4 illustrates the effect of different memristor non-idealities on the quality of the generated images and required number of the training iterations to achieve the high quality images produced by the generator. Figure 4(a) shows the effect of the limited number of stable resistive states in memristive devices on the quality of generated images. From Fig. 4(a), it can be observed that memristive devices with 64 or more resistive levels can be used without causing significant degradation of the image quality.

Figure 4(b)illustrates the effect of the memristor variability on the performance of the Generator. This includes random cell-to-cell variability following Gaussian distribution (the stochasticity of *R*_*ON*_/*R*_*OFF*_ values of the device in each memristor cell) and possibility of write/read error, when the final programmed value may have a deviation from the ideal case. The variation is resistive states in memristors follows as Gaussian distribution (explained in the Methods section). The results in Fig. 4(b) are shown for the memristive devices with 128 stable resistive states. The architecture can tolerate the distribution of memristive weights (represented as a conductance of the device) with the standard deviation of 0.04 from the ideal weight, and after *std* = 0.08 the image quality degrades significantly.

Figure 4(c) illustrates the effect of random failures of the memristive devices on the generated images. The device failure is introduced randomly considering three cases, when: (1) device is stack in *R*_*ON*_ state, (2) device is stack in *R*_*OFF*_ state and (3) complete failure of the device, when the current flow is disturbed. The device failure has a significant impact on the performance on the network, and the architecture can tolerate only up to 0.3–0.5% of device failures.

Figure 4(d) illustrates the effect of device aging^29,30^ on the performance of the architecture. The uniform aging of *R*_*ON*_ and *R*_*OFF*_ states was assumed (explained in Methods), where certain percentage of high and low resistive states is removed. The architecture can tolerate 2–4% of aging without the significant reduction of the quality of generated images.

Figure 4(e) shows how the variation in hardware and deviation from the ideal output affects the quality of the generated images. Random hardware noise was introduced to the outputs of all the activation functions as *y*_*n*_ = *y* × *R*_*d*_(1 − *x*/100, 1 + *x*/100), where *y* is an ideal output, *y*_*n*_ is a noisy output, *R*_*d*_(*a*, *b*) is a random uniform distribution with minimum value *a* and maximum value *b*, and *x* represents added noise in percentage. Figure 4(e) illustrates the effect on only hardware noise (left side) and the effect of hardware noise with memristor variation with *std* = 0.02 (right side). In the generated images without memristor variation, the generated numbers can still be recognized even with 40% of the noise in hardware, even though the generated images are noisy. However, in the experiment with both hardware variation and memristor variation, the quality of generated images significantly reduces after 10% of hardware noise.

Figure 4(f) illustrates the effect of the noise in the input images to the discriminator during training following random normal distribution on the quality of the generated images. Such noise in the input images may be a result of the non-idealities of the interface between the analog pixel sensor and the proposed architecture in the near-sensor processing. The noise is added according to the equation *z*_*n*_ = *z* + *R*_*d*_(−*x*/100, *x*/100), where *z*_*n*_ is the noisy image, *z* is an ideal input image, *x* is the added input noise in percentage considering that the image pixel values are normalized in the range of [0,1]. According to Fig. 4(f), the system can tolerate up to 10% of added random noise.

Finally, Fig. 4(g) illustrates the effect of number of training epochs on the generated image showing that 50 epochs, corresponding to maximum 3M update cycles of memristive devices, can produce good image quality (used in the calculated of required number of memristor update cycles).

  Figure 5 shows the quantitative analysis of the generated images represented by Frechet Inception Distance (FID) score^31^ calculated for 10,000 generated images compared to 10,000 randomly selected images from the training set of the MNIST database. Provided FID scores correspond to the generated images shown in Fig. 4. The meaning and calculation of the FID score is explained in Methods. The simulation results in Fig. 5(a) show that relatively low FID score for the architecture with limited number of resistive states can be achieved starting from 32 states. Figure 5(b–d) illustrate the calculated FID scores for variation in resistive states, device failure and aging, respectively. The dependence of FID score on memristor variation and percentage aging is close to linear. While, even insignificant percentage of the device failure in the system affects FID score and quality of generated images significantly. Figure 5(e) illustrates the effect of the hardware variation (noise) on the performance of the architecture without memristor variability and with memristor variability of *std* = 0.02. While for hardware variation of up to 35% the memristor variability (blue line) contributes significantly to the increase of FID score, the FID scores for the simulation with and without memristor variability become almost identical for large variation in hardware (after 35%). In addition, the effect of hardware variation cause smaller deterioration of the quality of generated images than the memristor variation for the given parameters. Figure 5(f) illustrates FID scores for noisy input images, where FID score increases significantly after 10% of the input noise, which correlates with the results illustrated in Fig. 4(f).

**Figure 5:** FID score for the simulation with (**a**) limited number of memristive levels (stable resistive states), (**b**) variability in memristive devices, (**c**) random device failures, (**d**) device aging, (**e**) hardware variation/noise, and (**f**) noise in images on the performance.

### Circuit level simulations

#### Circuit analysis

The circuit level simulations of transient and DC responses of individual AM-DCGAN components are shown in Fig. 6. For each circuit block, DC analysis, transient analysis, temperature analysis and Monte Carlo (MC) analysis for transistor geometry variation are performed. Temperature analysis is illustrated for the temperature range from −15 °*C* up to 65 °*C*. MC analysis is shown for the 10% random variation of CMOS transistor length *L*, which effects the performance of the circuit the most.

**Figure 6:** Circuit analysis of GAN components from Fig. 2. DC, transient analysis, temperature analysis and Monte Carlo variation (10%) of transistor length L for (**a**) hyperbolic tangent, (**b**) Rectifier Linear Unit (ReLU), (**c**) Leaky ReLU, (**d**) current to voltage converter (IVC), (**e**) operational amplifier (OpAmp), (**f**) weight sign switch circuit, (**g**) control switch for the crossbar, and (**h**) Sample and Hold (SH) circuit.

Figure 6(a) presents the simulation results of the hyperbolic tangent activation function circuit, where DC response is compared to an ideal hyperbolic tangent function. The temperature affects the threshold of hyperbolic tangent, as well as the variation in *L* shown in the MC analysis. The simulation of the Rectifier Linear Unit (ReLU) circuit in Fig. 6(b) shows the operation region to be approximately [−2.5 V, 2.5 V]. The temperature variation effect on the DC characteristics of the proposed ReLU circuit is negligible, as the ReLU threshold varies withing [−15 *mV*, 30 *mV*] instead of ideal 0*V* output. The 10% *L* variation causes the threshold shift of up to 70 *mV*. The simulation results for LeakyReLU circuit are shown in Fig. 6(c). The temperature and *L* variations for LeakyReLU are similar to the ones in the ReLU circuit.

Figure 6(d) presenting the simulation results of the current to voltage converter (IVC) show the results of both the inverted *V*_*inv*_ and non-inverted *V*_*outIVC*_ outputs. The simulation results of the operational amplifier (OpAmp) circuit from Fig. 6(e) lead to a slew rate of 3.7 × 10^9^ *V*/*s* and unity gain bandwidth of 2.4 *GHz*. This allows for high speed operation of the proposed AM-DCGAN circuit. Figure 6(f) presents the analysis of weight sign switch (WSS) circuit depicting their ability to change or retain the sign of the input signal. The temperature analysis of the OpAmp and OpAmp-based circuits, such as IVC and WSS, illustrates that the temperature effect on the performance of the circuits are negligible. The MC analysis of the OpAmp circuit shows that the output vary withing the range of [−0.2 *V*, 0.2 *V*] with the 10% of *L* variation, and this variation is increased in the OpAmp-based circuits, where two OpAmps and additional circuit components, such as inverters and transmission gates, are used.

Figure 6(g) illustrates the simulation results for control switch for the crossbar columns in ON and OFF states. The temperature variation does not affect the performance of the switch. The variation of transistor length *L* does not cause the significant deviation from the ideal output. Figure 6(h) illustrates the performance analysis of the SH circuit, where first two graphs show the clock signal *V*_*clk*_ and corresponding input voltage and sampled output voltage. The temperature variation does not affect the performance of SH circuit, as well as *L* variation.

Table 1 shows maximum power consumption, on-chip area and delay in various circuit components of the system. We designed the circuit using a stable 180 nm CMOS technology to prove that GAN circuit can work with memristive devices. Knowm MSS (Multi-Stable Switch) model is used to simulate the WOx memristive devices^32^.This however, has led to high power consumption and can be reduced by using smaller geometry processes. The on-chip area of CMOS part of the complete Generator configuration with 3 layers containing [128, 64, 1] filters, input noise size of 7 × 7 and output image size of 28 × 28 is 0.581 *mm*^2^. The overall delay for forward propagation in the Generator circuit with 3 layers is about 0.68 *ns*. On the other hand, the delay in the Discriminator circuit with 3 convolutional and 2 dense layers is 0.122 *μs*. This is due to the sequential processing in the crossbar columns in the dense layers. Hence, after training, the Generator circuit can have high performance speed, as the processing is performed in analog domain and analog to digital conversion stage does not limit the processing speed by the sampling rate of ADCs and DACs. Nevertheless, if it is desired to reduce power consumption, this fast speed can be compromised introducing sequential processing in the layers.

**Table 1:** On-chip area, maximum power consumption and delay calculation for the circuit blocks used in GAN architecture.

Circuit block	Power consumption (*mW*)	On-chip area (*μm*^2^)	Delay (*ps*)
ReLU	0.112	23.659	322
LeakyReLU	2.155	35.809	420
Hyperbolic tangent	0.112	0.259	36
Difference amplifier	37.625	54.432	540
Operational amplifier	8.261	44.712	620
Control switch	11.200	10.840	175
IVC	72.036	96.714	454
Weight sign switch	41.449	117.331	251
Sample and Hold circuit (without buffers)	0.0005	7.4838	60
Voltage buffer	42.000	44.712	150

#### CMOS scaling

Scaling of the proposed architecture for smaller CMOS technology allows to improve power consumption and on-chip area of the system. We show the comparison of system components, filters and crossbars designed in 45 nm CMOS technology to 180 nm CMOS circuits. The simulations were performed using 45 nm CMOS PTM models^33^.

Table 2 shows the changes in the performance metrics, such as power consumption, on-chip area, circuit delay, temperature and transistor length variation effects, due to scaling down of the circuits to 45 nm with *V*_*DD*_ = 1*V* for separate circuit components and for filters with activation functions and dense layer crossbar. In general, the power consumption and on-chip area are significantly improved, however, the temperature variation and transistor length *L* variation of the circuits designed 45 *nm* cause more significant output variation than for 180 *nm* CMOS technology. The delay of the circuits is affected by the used transistor length *L* in the design. In the circuits with minimum *L* = 45 *nm*, the delay is decreased, comparing to 180nm circuits; however the delay increases if the circuit length is set to *L* = 90 *nm*.

**Table 2:** Scaling of the design for 45 nm CMOS technology and comparison to 180 nm.

Component		Power (mW)	Power	Area (*μm*^2^)	Area change	Delay (ps)	Delay change	T∘C var. range (offset)	T∘C var. change	L var. (offset)	L var. change
**Separate circuit components**											
ReLU		0.053	↓53%	1.479	↓94%	100	↓70%	±60 *mV*	↑60%	±0.2 *V*	↑60%
LeakyReLU		2.050	↓5%	2.037	↓94%	80	↓81%	±60 *mV*	↑65%	±0.2 *V*	↑60%
Tanh		0.017	↓85%	0.062	↓76%	64	↑44%	±80 *mV*	↑50%	±0.3 *V*	↑67%
Opamp	*L* = 45 *nm*	2.290	↓72%	2.724	↓94%	160	↓74%	±0.1 *V*	↑50%	±0.25 *V*	↑25%
	*L* = 90 *nm*	0.798	↓90%	5.448	↓88%	650	↑5%	±12 *mV*	↓88%	±50 *mV*	↓75%
WSS circuit	*L* = 45 *nm*	2.719	↓93%	8.744	↓92%	650	↑61%	±10 *mV*	↑90%	large variation^*3^	
	*L* = 90 *nm*	1.320	↓97%	11.468	↓90%	4000	↑94%	±0.1 V^*2^		±0.3 V^*4^	—
CS circuit		11.00^*1^	↓2%	0.675	↓94%	120	↓31%	no variation		±1mA^*5^	↑50%
**Component**				**Power (mW)**	**Area** (***μm***^**2**^)	**Delay (ns)**	Output errors^*6^				
**Filters and crossbars (comparison of 180 nm and 45 nm CMOS circuits)**											
Convolutional filter with LeakyReLU			180 *nm*	40.16	177.72	1.28	Diff.amplifier: 0.9 *mV*			ReLU: 0 *mV*	
			45 *nm*	1.63	10.84	1.88	Diff.amplifier: 0.24 *mV*			ReLU: 0.2 *mV*	
Convolutional filter with Tanh			180 *nm*	40.08	142.17	1.15	Diff.amplifier: 0.9 *mV*			Tanh^*7^: 0.3 *mV*	
			45 *nm*	1.38	8.86	1.80	Diff.amplifier: 0.17 *mV*			Tanh^*7^: 0.2 *mV*	
Dense layer crossbar with LeakyReLU			180 *nm*	441.9	1454	1.45	WSS(i): 1.04 *mV*	WSS(n): 0.76 *mV*	CS: ~0 *mV*	IVC: 0.3 *mV*	L.ReLU: ~0 *mV*
			45 *nm*	15.53	131.9	6.25	WSS(i): 2.15 *mV*	WSS(n): 0.63 *mV*	CS: ~0 *mV*	IVC: 0.8 *mV*	L.ReLU: ~0 *mV*

^*1^Depends on the current; ^*2^for input voltages >0.8 V; ^*3^distortion of the output; ^*4^can cause distortion of the output in rare cases; ^*5^only for the input >∣8 *mA*∣; ^*6^example for particular case; ^*7^for small input (error in the slope; Abbreviations: L.ReLU-LeakyReLU, WSS(i/n)- inverted/non-inverted output of WSS).

When scaling down, the operation range of the ReLU and LeakyReLU circuits decreased to [−1.2 *V*, 1.2 *V*] due to the decrease of *V*_*DD*_. In addition, for the small input voltages [−8 *mV*, 8 *mV*], the offset of 2 *mV* occurs, which can be improved by optimizing the inverters *M*_1_ − *M*_4_. In the Tanh circuit, there is a small offset (maximum 0.1 *V*) in the DC response and the slight change in the slope for the input voltage of 0.1 *V* − 0.6 *V*, which can be further improved by optimizing the circuit parameters. If the OpAmp circuit is scaled to the minimum length *L* = 45 *nm*, the circuit performance is affected by the temperature and *L* variation, also it does not reach *V*_*DD*_ = 1 *V* (only 0.8 *V*) in a closed loop configuration, while the delay is reduced. Therefore, the performance of the OpAmp with *L* = 90 *nm* is shown. Such OpAmp is more stable and accurate, comparing to the one with *L* = 45 *nm*, however the increase in *L* affects the dynamic behavior of the circuit and causes the output delay. In the scaling of the WSS circuit, *R*_11_ and *R*_12_ are increase to 2 *k*Ω to improve the performance. If the OpAmp with *L* = 45 *nm* is used in WSS, the operation range is reduced and the variation in temperature and *L* can cause the distortion of the output. Therefore, the OpAmp with *L* = 90 *nm* is more effective for such circuit, however 4 *ns* is required for the circuit to fully stabilize.

The second part of Table 2 compares the performance of the convolutional filters and dense layer crossbar and processing circuits in terms of power consumption, on-chip area, total delay and errors at different parts of the circuit. The convolutional filters were simulated with 10 positive and negative weights followed by the difference amplifier and LeakyReLU or Tanh circuits. The dense layer crossbar was simulated with 9 × 9 memristors in both main and sign crossbar, 9 WSS circuits, CS, IVC and LeakyReLU circuits. The *R*_8_ − *R*_10_ resistance values for convolutional filters and *R*_13_ − *R*_15_ for IVC in the dense layer have been increase to 1 *k*Ω to avoid the impact of the processing circuits on the memristive crossbar. Overall, the power consumption and on-chip area decrease significantly for 45 *nm* CMOS technology, however, the delay increases. The output errors vary for different components of the system. For successful scaling for the design, the trade-off between processing speed affected by the circuit delay and on-chip area and power consumption should be found.

#### Memristor variability effect

Variability and non-idealities of memristive devices can deteriorate the performance of the architectures. Hence, Monte Carlo simulations were also performed to understand the operational limits of the circuit. As actual memristor variations are not very well known, we used large conservative estimates of 10% and 30% variations in memristor performances. A typical Generator circuit with 2 deconvolutional layers with ReLU activation functions and one final layer with hyperbolic tangent was used. Figure 7(a–f) shows these results. The first row (Fig. 7(a,b)) compares the performance of the circuit with ideal response showing very little absolute error in both Relu as well as tanh output nodes. The second and third row of Fig. 7 (Fig. 7(c–f)) show results of introducing variability at 10% and 30% respectively. It can be observed that the tanh layer has higher sensitivity to memristor variability. This is expected as being the output layer, it also accumulates errors from all previous layers. The output spikes in the timing diagram are caused by the delay of inverters in ReLU circuit and can be compensated with additional circuit components.

**Figure 7:** Output of the Generator (**a**–**f**): (**a**) ideal vs circuit output after ReLU, (**b**) after hyperbolic tangent in the last layer. Variability analysis of memristive devices: (**c**,**d**) effect on ReLU and hyperbolic tangent output for 10% variability in memristive devices; (**e,f**) 20% variability. (**g**–**k**) Errors caused by the variabilities in memristive weights in the Discriminator (CNN): (**g,h**) error in the output of the convolutional filter ((**g**) particular example of two separate filters, and (**h**) average of 10 random cases with 10 iterations), (**i**) error in the mean filter, (**j**) error in the dense layer input after, and (**k**) error in the output current in the dense layer.

Figure 7(g–k) illustrates the simulation of variability analysis in convolutional and dense layers of a small scale CNN (the Discriminator) for forward propagation during training with different percentage of memristor variability (from 0% to 40%). The simulation was performed for 10 particular cases with 10 random iterations of the variation in memristor values, and the average value is reported for 1st convolutional filter output, mean filter output, dense layer input and dense layer output (Fig. 7(h–k)). The results for the 1st convolutional filter output variation show that the error for 30% is 2–3% less than the error for 40% memristor variation. This is due to the testing of only few particular random cases of memristor variation and averaging of the final error results. Overall, the output errors for 30% and 40% variation are similar, as illustrated by the example in Fig. 7(g), where the output variation of two different convolutional filters is shown. As the signal propagates through the memristive levels, the errors at the output of each stage increase and accumulate for the next stage.

#### Training time and power

Based on Fig. 4(e), we also calculated the time and power required for the update (training) cycle. We consider WO_*x*_ memristive devices, with *R*_*ON*_ = 40 *k*Ω and *R*_*OFF*_ = 250 *k*Ω, threshold voltage 0.8 *V*, write voltage 1 *V* and different “write” times. These were used in a three layer Generator and Discriminator architectures with 1.7 million memristive weights for 50 epochs. 60,000 MNIST images of size 28 × 28 were used. Furthermore, a maximum of 128 convolutional filters of the size of 5 × 5 are used. These results for different ways of parallel and sequential update of memristors in the architecture are shown in Table 3. The training time per epoch and average power per computation is reported. Considering the number of required update cycles for memristive devices from Table 3 and Fig. 4(c), the memristor endurance for on-chip training of such networks may be a problem. In such cases, one may consider the use of AM-DCGAN for partial image-generation and network training. The software or microprocessor based pre-training up to certain accuracy followed by complete hardware-based training can be used to improve the learning speed of AM-DCGAN.

**Table 3:** Training time per epoch for memristors with different time required for write cycles (10 *ns*, 100 *ns* and 1000 *ns*) and average power consumption per neural computation.

Update Configuration	Power (W)			Training time (s)	
	max	min	10 ns	100 ns	1000 ns
Parallel update of independent columns in layers and independent layers	0.28 *μ*	47.08 *n*	0.47	4.71	47.10
Update of memristors in 4 cycles of independent layers in series (rows and columns)	2.52 *μ*	0.408 *μ*	0.014	0.144	1.44

## Discussion and Conclusion

This paper proposes the first implementation of fully analog memristive hardware implementation of AM-DCGAN. The practical aspects such as endurance, limitations on conductive levels, and circuit parasitics from wires and devices were included in the design and simulations. The system remains stable for conductance variation up to *std* = 0.04 with 128 conductance levels, and inference performance substantially degrades at *std* = 0.08. The system can tolerate up to 4% of memristor aging and up to 0.3–0.5% of device failures in the proposed architecture. The hardware variation (noise) reduces the quality and adds noise to the generated images, while the hardware variation up to 10% with memristor variability can still be tolerated. Up to 10% of noise in the input images, that can be the result of the interface between image sensor and the proposed circuit in near-sensor processing, can also be tolerated. By treating the memristive neural networks as hardware subroutines, it is possible to develop an analog system that can speed up complex neural computing for near-sensor data processing of GAN. The main advantages of AM-DCGAN are small on-chip area and possibility to implement it on edge devices and integrate directly to analog sensors to process information in real time and speed up the training. The WO_*x*_ memristive devices are compatible with 180 *nm* CMOS process^11^, and the proposed CMOS-memristive system can be fabricated using Back-End-of-Line (BEOL) process^34^ placing the memristive crossbars on top of the CMOS circuits.

In this work, only basic non-idealities of memristive devices, which traditionally affect the performance of the neural networks significantly, have been considered. While the memristor variation effect shown in the simulation results illustrates the worst case scenario, where for *std* > 0.04 even the highest and lowest memristive states can correlate, and the aging simulation cause some of the states to disappear, the effect of non-linearity of memristor programming and non-linear distribution of resistive states in the particular devices can be studied further.

The design of the control circuit and overall chip implementation of the proposed GAN are still open research problems and may be considered in future works. In addition, the implementation of more complex analog GAN architecture with max-pooling, normalization and an on-chip training unit for generation of more complex images is an open problem that can be addressed in future. While, MNIST handwritten digits generation of the size of 28 × 28 illustrates that memristive devices with variabilities and limited number of stable resistive states can still be used for analog GAN implementation, more complex cases with large image, and in turn increased hardware complexity, should be considered as a research direction for the further implementations of analog memristor based GAN architectures.

## Methods

### Technology, models and tools

The system level simulation for image generation was performed in Python, considering the outputs and non-idealities of the circuits verified in SPICE. The circuit level simulations were performed in SPICE using 180 nm CMOS technology and Knowm MSS (Multi-Stable Switch) memristor model^32,35^ based on the parameters of WO_*x*_ memristive devices^19,36^. In this model, the current of the device is described by two components, memory-dependent current *I*_*m*_ and Schottky diode current *I*_*s*_^37^, shown in Eq. (2).

2 $$I=\phi {I}_{m}(V,t)+(1-\phi ){I}_{s}(V)$$

The Schottky current *I*_*s*_ induced by the metal-semiconductor junction in memristive device and can be represented as ${I}_{s}={\alpha }_{f}{e}^{{b}_{f}V}-{\alpha }_{r}{e}^{-{b}_{r}V}$, and the parameter *ϕ* ∈ [0, 1] shows the impact on this current on the device. The parameters *α*_*f*_, *β*_*f*_, *α*_*r*_, *β*_*r*_ are positive device specific constants describing an exponential behavior of *I*_*s*_, which are different for each memristor material. The conductance of the device is represented as a total conductance of *N* metastable switches. The memory-dependent current *I*_*m*_ can be represented as *I*_*m*_ = *V*(*G*_*m*_ + Δ*G*_*m*_), where *G*_*m*_ is a total memristor conductance over *N* metastable switches and Δ*G*_*m*_ is a change in conductance relying on the distributions *P*_*A*_ and *P*_*B*_^37^. The distributions *P*_*A*_ and *P*_*B*_ are the probability of transition between *A* and *B* states are shown in Eqs. (3) and (4), where $\beta ={V}_{T}^{-1}$ is a thermal parameter, and *α* = Δ*t*∕*t*_*c*_. The parameter Δ*t* is time step ratio, and *t*_*c*_ is a time scale of the device^32^.

3 $${P}_{A}=\alpha \frac{1}{1+{e}^{\beta (V-{V}_{A})}}=\alpha \Gamma (V,{V}_{A})$$

4 $${P}_{B}=\alpha (1-\Gamma (V,-{V}_{B}))$$

The parameters of the applied WO_*x*_ memristors are the following: *R*_*ON*_ = 40 *k*Ω, *R*_*OFF*_ = 250 *k*Ω, *V*_*A*_ = 0.8 *V*, *V*_*B*_ = 1 *V*, *t*_*c*_ = 0.8, *ϕ* = 0.55, *α*_*f*_ = 10^−9^, *β*_*f*_ = 0.85, *α*_*r*_ = 22 × 10^−9^, *β*_*r*_ = 6.2^32^.

### FID score calculation

The calculation of FID score is shown in Eq. (5)^31,38^, where (**m**, **C**), (**m**_**w**_, **C**_**w**_) are feature-wise image mean and covariance matrices of real and generated images, *Tr* is a sum all elements of the image matrix along the main diagonal.

5 $${d}^{2}(({\bf{m}},{\bf{C}}),({{\bf{m}}}_{{\bf{w}}},{{\bf{C}}}_{{\bf{w}}}))=\parallel {\bf{m}}-{{\bf{m}}}_{{\bf{w}}}{\parallel }_{2}^{2}+Tr\left({\bf{C}}+{{\bf{C}}}_{{\bf{w}}}-2\sqrt{{\bf{C}}{{\bf{C}}}_{{\bf{w}}}}\right)$$

The FID scores for memristor variation and device failure in Fig. 5 are calculated as an average of 10 random cases of different variabilities and device failures.
